The article "Changes in Levels of Homocysteine and C-Reactive Protein in Patients with Alzheimer's Disease and Their Correlation with Cognitive and UPDRS Functions" was retracted in 2023. Reasons: signs of a paper mill; suspected computer-generated content; unreliable results or conclusions; concerns about the data.

# Changes in Levels of Homocysteine and C-Reactive Protein in Patients with Alzheimer's Disease and Their Correlation with Cognitive and UPDRS Functions

**DOI:** 10.1155/2022/4661687

**Published:** 2022-09-22

**Authors:** Xiaolin Gu, Tingting Li, Junzeng Si, Longfei Gao, Yan Li, Aiqin Qi

**Affiliations:** Department of Neurology, Jinan People's Hospital Affiliated to Shandong First Medical University, Jinan 271100, China

## Abstract

**Objective:**

To investigate the changes in the levels of homocysteine (Hcy) and C-reactive protein (CRP) in patients with Alzheimer's disease (AD) and analyze their correlation with cognitive and UPDRS functions.

**Methods:**

A total of 50 patients with AD admitted to our hospital from January 2020 to March 2022 were selected into the research group, and 50 healthy subjects were selected as the control group. The levels of Hcy and CRP of the two groups were analyzed, and the patients' cognitive functions were evaluated with the Mini-Mental State Examination (MMSE) score and UPDRS function scoring. The correlation between the changes in levels of Hcy and CRP, and cognitive and UPDRS functions in the two groups was compared and analyzed.

**Results:**

The levels of Hcy and CRP of the research group were higher than those of the control group, with statistical significance (*P* < 0.05). The following were evaluated for the scoring of patients' cognitive functions in the research group: orientation, attentional computation, short-term memory, language ability, visuospatial ability, instant memory, and MMSE total score, all of which were lower than those in the control group, with statistical significance (*P* < 0.05). UPDRS I, UPDRS, UPDRS, and total UPDRS score in the research group were higher than those in the control group, with statistical significance (*P* < 0.05). In the research group, the higher the Hcy level, the lower the MMSE score, with a negative correlation (*P* < 0.05), and the higher the Hcy level, the higher the UPDRS score, with a positive correlation (*P* < 0.05). And, the higher the CRP level, the lower the MMSE score, with a negative correlation (*P* < 0.05); the higher the CRP level, the higher the UPDRS score, with a positive correlation (*P* < 0.05).

**Conclusion:**

Compared with the health subject group, the levels of Hcy and CRP were higher in patients with AD, and their changes had a negative correlation with cognitive functions in patients with AD, and a positive correlation with UPDRS in patients with AD, with high clinical values in evaluating cognitive and UPDRS functions.

## 1. Introduction

Alzheimer's disease (AD) is a relatively common neurological disease in clinical treatment. Patients are mainly accompanied by progressive cognitive dysfunction, behavioral dysfunction, and other clinical manifestations, with the annually increasing incidence currently [1]. The pathogenesis of AD is still under study, and no specific treatment regimen has been found for this disease in clinics. Therefore, it is necessary to make an early diagnosis and give corresponding intervention measures to improve the prognosis and quality of life of patients, and relieve the economic pressure and care burden of their families [2, 3]. During the process of clinical diagnosis and evaluation, the use of high-sensitivity, scientific, and accurate serological indicators is of positive significance to the treatment of patients and the quality assessment of their prognosis [4]. As one of the conventional indicators to evaluate the inflammatory state, the increase of C-reactive protein (CRP) concentration in the body indicates the aggravation of the inflammatory state in the body, and the change of its level is positively correlated with the inflammatory state in the body [5]. Homocysteine (Hcy) is one of the indexes for the routine evaluation of vascular lesions in patients, which can clearly analyze the situation of atherosclerosis in patients, so as to evaluate the endovascular atherosclerosis in patients. According to the research materials [6, 7], the changes in the concentration of CRP and Hcy have the correlation with cognitive dysfunction in patients. However, there are rare research materials in clinics. In this study, the correlation between the concentrations of CRP and Hcy, and patients' cognition and UPDRS functions was analyzed in patients with AD and healthy controls at the same time, and the desired effect was achieved, which was especially reported as follows.

The article "Changes in Levels of Homocysteine and C-Reactive Protein in Patients with Alzheimer's Disease and Their Correlation with Cognitive and UPDRS Functions" was retracted in 2023. Reasons: signs of a paper mill; suspected computer-generated content; unreliable results or conclusions; concerns about the data.

## 2. Materials and Methods

### 2.1. General Information

Fifty patients with AD admitted to our hospital from January 2020 to March 2022 were selected as the research group, including 24 males and 26 females, aged from 65 to 80 years, with a mean age of 70.67 ± 2.10 years, who had AD for 2∼10 years, with the mean disease course of 5.48 ± 0.23 years. And, 50 health examinees were selected as the control group in the same period, including 25 males and 25 females, aged from 65 to 79 years, with the mean age of 70.37 ± 2.23 years. There was no significant difference in gender ratio and age between the two groups (*P* > 0.05), indicating comparability. The inclusion criteria are as follows: the participants in the study were aged from 65 to 80 years, without organic lesions in the heart, liver, and kidney, who were informed about this study and signed the informed consent documents. The study has been reviewed by the ethics committee of the hospital. The exclusion criteria are as follows: both groups excluded the patients who were unwilling to participate or did not actively cooperate, those with other mental system disorders or cognitive dysfunction, and those with secondary admission for diagnosis or treatment. Patients with thyroid disease, obesity, liver, kidney, and other organic diseases, those who were confirmed as other brain diseases by head CT or MRI diagnosis, and those without infection or tissue damages within 2 weeks were excluded.

### 2.2. Methods

The patients in both groups were detected for CRP and Hcy, which was conducted as follows: Hcy detection in serum: 5 ml of fasting venous blood (fasting for 12 h or longer) was collected from the subjects in the two groups in the morning by vacuum vasculature, which was then centrifuged at 3000 r/min for 15 min. An appropriate amount of serum was taken and stored aseptically at −20°C. Hcy was detected by fluorescence polarization immunoassay with chemiluminescence immunoassay equipment and professional reagents produced by Siemens in strict accordance with the instructions. The testing process must be performed according to the requirements of the kit. The remaining serum was tested for CRP by the immunoscattering turbidimetry method, which was conducted by the BNProSpec automatic immunoisolated turbidity equipment and professional supporting reagents produced by Siemens in the United States in strict accordance with the instructions.

### 2.3. Observation Indexes

The levels of Hcy and CRP in the two groups were analyzed, both of which were also compared between the two groups.

The cognitive functions of the two groups were determined and evaluated with the MMSE scale, mainly from the aspects including orientation, attention to calculation, short-term memory, language ability, visual spatial power, and instant memory, and the total MMSE score was recorded.

UPDRS functions of both the groups were determined and evaluated with the UPDRS score, mainly including the UPDRS I score (mainly from spirit, behavior, and emotion), UPDRS II score (mainly from the daily life of the patients), and UPDRS III score (mainly from the motor ability of the patients).

In the research group, the patients with an MMSE score of 21 or more had mild cognitive dysfunction, those with a score of 10∼20 had moderate cognitive dysfunction, and those with a score of 9 or less had severe cognitive functions. According to the score, the correlation between the levels of Hcy and CRP and the MMSE score of patients with different AD types was analyzed.

During the scoring of UPDRS, the total score of 0∼20 is classified as mild dysfunction, that of 21∼40 as moderate dysfunction, and that of 41∼60 as severe dysfunction. According to this score, the correlation between the levels of Hcy and CRP, and the MMSE score of patients with different AD types was analyzed.

The article "Changes in Levels of Homocysteine and C-Reactive Protein in Patients with Alzheimer's Disease and Their Correlation with Cognitive and UPDRS Functions" was retracted in 2023. Reasons: signs of a paper mill; suspected computer-generated content; unreliable results or conclusions; concerns about the data.

### 2.4. Statistical Analysis

The data were analyzed with the statistical software SPSS20.0. Measurement data were expressed with $\bar{x}$ ± *s*, the *t*-test was used for the comparison between the two groups. Enumeration data were expressed with the rate and tested with *x*^2^. *P* < 0.05 was considered as a statistically significant difference.

## 3. Results

### 3.1. Comparison of Levels of Homocysteine and C-Reactive Protein between the Two Groups

The patients in the research group had higher levels of Hcy and CRP than those in the control group, which was statistically significant (*P* < 0.05), as shown in Table 1.

### 3.2. Comparison of Cognitive Function Scores between the Two Groups

The patients' scores of cognitive functions in the research group, including orientation, attention to calculation, short-term memory, language ability, visual spatial power, instant memory, and the total MMSE score, were all lower than those in the control group, which were statistically significant (*P* < 0.05), as shown in Table 2.

### 3.3. Comparison of UPDRS Scores of the Samples

The total scores of UPDRS I, UPDRS, UPDRS, and UPDRS of the patients in the research group were higher than those in the control group, which was statistically significant (*P* < 0.05), as shown in Table 3.

### 3.4. Correlation Analysis of Patients' Hcy with Cognitive Functions

For the patients in the research group, the higher the Hcy level, the lower the MMSE score, which was negatively correlated (*P* < 0.05), but the higher the Hcy level, the higher the UPDRS score, which was positively correlated (*P* < 0.05), as shown in Tables 4 and 5.

### 3.5. Correlation Analysis of Patients' CRP with Cognitive Functions

For the patients in the research group, the higher the CRP level, the lower the MMSE score, which was negatively correlated (*P* < 0.05), but the higher the CRP level, the higher the UPDRS score, which was positively correlated (*P* < 0.05), as shown in Tables 6 and 7.

## 4. Discussion

AD is also known as senile dementia in clinical treatment, which is a common degenerative brain lesion. Patients who have got this disease will be accompanied by progressive memory decline, cognitive dysfunction, and abnormal behavioral ability, which has a serious impact on patients' life, health, and safety [8, 9]. AD can last for about 3–20 years, and can also increase the financial burden and care burden of the society and families. With the aging of the domestic population, the number of patients with AD is increasing [10]. According to the incomplete statistics on this disease in western developed countries, more than 10% of the elderly people have got AD, and the incidence of the elderly groups aged 85 years or above is as high as 20∼48%. The domestic survey of AD has also shown that the incidence of this disease has surpassed that of western developed countries [11]. It is expected that there will be more than 60 million patients having got AD by 2030 in the world, and at that time, this disease will become one of the serious diseases threatening the safety of humans' life and health.

The article "Changes in Levels of Homocysteine and C-Reactive Protein in Patients with Alzheimer's Disease and Their Correlation with Cognitive and UPDRS Functions" was retracted in 2023. Reasons: signs of a paper mill; suspected computer-generated content; unreliable results or conclusions; concerns about the data.

The internal brain tissues of patients with AD are associated with unconventional protein deposition reactions, which mainly include extracellular amyloid polypeptide deposition and intracellular nerve fiber tangle reaction [12]. The research materials showed that [13], in AD, inflammation occurs in the lobes and hippocampus of the brain, resulting in age-like blotches. In addition, the activation of microglia and astroglia in the brain plays a certain role in the occurrence and development of AD in patients. Therefore, it is of great importance for the way to use high-sensitivity, scientific, and accurate indexes to assess the early diagnosis, prognosis, and treatment of patients with AD. A small number of studies have stated that patients with AD have an internal immune inflammatory reaction during the development of the disease, and Hcy and CRP are closely involved in the pathological changes of patients, with a certain effect [14].

Hcy is a kind of sulfur amino acid, which is one of the products of the demethylation reaction in methionine metabolism. Hcy that cannot continue to be metabolized to cysteine will be accumulated in the body. Over-accumulation of Hcy can block the metabolic level of prostacyclin in the body, so that the LDL level continues to increase, which will affect the function of the vascular wall, causing damage to the wall of the tube, accelerating the rate of thrombosis, intensifying the blood clotting response, and finally, patients will be prone to atherosclerotic lesions. After consulting domestic research materials, it was found that a high Hcy level will increase the cerebrovascular endothelial damage and prethrombotic status in patients with AD, and other materials also indicate that a high Hcy level in the body will inhibit the activity of lysyl oxidase itself in the vascular endothelial cells, generating superoxide anions and derivative substances such as nitric oxide nitrite in the body, so that the body will be accompanied by damage to the nitric oxide pathway, and may have an excessive oxidative stress response [15]. CRP is a special protein synthesized and secreted by liver tissues, which is widely used in the evaluation of inflammatory response. In patients with AD complicated with different degrees of inflammatory reactions, inflammatory factors will accumulate in the tissues around the lesions, affect the metabolism of healthy cells, cause death of numerous healthy cells, and the functions of cranial neurons themselves will be seriously affected; therefore, the degree of cognitive dysfunction in patients with AD can be assessed by CRP. The data of this study showed that the levels of Hcy was higher in patients in the research group than those in the control group, with statistical significance (*P* < 0.05), indicating that compared with healthy people, patients with AD tend to have increased levels of Hcy and CRP. The patients' scores of cognitive functions in the research group, including orientation, attention to calculation, short-term memory, language ability, visual spatial power, instant memory, and the total MMSE score, were all lower than those in the control group, which were statistically significant (*P* < 0.05), and the total scores of UPDRS I, UPDRS II, UPDRS III, and UPDRS of the patients in the research group were higher than those in the control group, which was statistically significant (*P* < 0.05). The results suggest that the patients with AD have more obvious cognitive dysfunction; in addition, the patients' mental, emotional, daily life activities, motor function indexes, and other indexes also changed significantly. For patients in the research group, the higher the Hcy level, the lower the MMSE score, showing a negative correlation (*P* < 0.05), but the higher the Hcy level, the higher the UPDRS score, showing a positive correlation (*P* < 0.05). In the research group, it was also found that the higher the CRP level, the lower the MMSE score, showing a negative correlation (*P* < 0.05), but, the higher the CRP level, the higher the UPDRS score, showing a positive correlation (*P* < 0.05). The results indicate that the two indexes are specific for patients' cognitive functions, including spirit, emotion, daily life activities, and motor function, and can be used as a clinical diagnostic basis and key indexes to evaluate the quality of prognosis, with the positive significance for the diagnosis and treatment of the disease and the prognosis of patients.

The article "Changes in Levels of Homocysteine and C-Reactive Protein in Patients with Alzheimer's Disease and Their Correlation with Cognitive and UPDRS Functions" was retracted in 2023. Reasons: signs of a paper mill; suspected computer-generated content; unreliable results or conclusions; concerns about the data.

In conclusion, compared with the health examinees, patients with AD have higher levels of Hcy and CRP, and the changes of levels of these two indexes are negatively correlated with cognitive functions, and positively correlated with the UPDRS score. Therefore, the two indexes have high clinical application values in evaluating cognitive and UPDRS functions of patients with AD.

## Figures and Tables

**Table 1:** Comparison of levels of homocysteine and C-reactive protein between the two groups ($\bar{x}$ ± *s*).

Group	Number of patients	Hcy (umol/L)	CRP (mg/ml)
Control group	50	3.37 ± 0.76	1.29 ± 0.23
Research group	50	18.76 ± 2.17	5.21 ± 1.17
*T*	—	47.330	23.246
*P*	—	<0.001	<0.001

**Table 2:** Comparison of cognitive function scores between the two groups ($\bar{x}$ ± *s*).

Group	Number of patients	Orientation	Attention to calculation	Short-term memory	Language ability	Instant memory	Visual spatial power	Total MMSE score
Control group	50	4.86 ± 1.24	4.69 ± 1.24	4.91 ± 1.12	4.68 ± 0.48	4.48 ± 1.09	4.32 ± 0.65	28.65 ± 3.25
Research group	50	3.08 ± 0.93	1.26 ± 0.53	1.11 ± 0.42	3.21 ± 0.65	2.24 ± 0.69	0.91 ± 0.23	12.26 ± 2.12
*t*	—	8.120	17.985	22.464	12.864	12.278	34.971	29.867
*P*	—	<0.001	<0.001	<0.001	<0.001	<0.001	<0.001	<0.001

**Table 3:** Comparison of patients' UPDRS scores ($\bar{x}$ ±*s*).

Group	Number of patients	UPDRS I	UPDRS II	UPDRS III	Total UPDRS score
Control group	50	1.02 ± 0.22	5.42 ± 1.28	10.89 ± 1.23	12.34 ± 2.17
Research group	50	2.35 ± 0.50	15.87 ± 3.29	30.28 ± 5.29	45.29 ± 10.28
*T*	—	16.656	20.931	25.245	22.176
*P*	—	<0.001	<0.001	<0.001	<0.001

**Table 4:** Correlation analysis of patients' Hcy with MMSE scores ($\bar{x}$ ± *s*).

Class	Number of patients	Hcy (umol/L)
Mild cognitive dysfunction (MMSE score ≥21)	15	16.78 ± 0.79
Moderate cognitive dysfunction (MMSE score of 10–20)	12	20.37 ± 3.49^a^
Severe cognitive dysfunction (MMSE score ≤9)	23	26.98 ± 4.39^ab^

*Note.* compared with patients with mild cognitive dysfunction, ^*a*^*P* < 0.05; compared with patients with mild and moderate cognitive dysfunction, ^b^*P* < 0.05.

**Table 5:** Correlation analysis of patients' Hcy with UPDRS scores ($\bar{x}$ ± *s*).

Class	Number of patients	Hcy (umol/L)
Total UPDRS score of 0∼20	12	17.93 ± 3.19
Total UPDRS score of 21∼40	17	22.17 ± 2.19^a^
Total UPDRS score of 41∼60	21	27.09 ± 3.29^ab^

*Note.* compared with patients with a total UPDRS score of 0∼20, ^a^*P* < 0.05; compared with the patients with a total score of 21∼40 and 41∼60, ^b^*P* < 0.05.

**Table 6:** Correlation analysis of patients' CRP with MMSE scores ($\bar{x}$ ± *s*).

Class	Number of patients	CRP (mg/ml)
Mild cognitive dysfunction (MMSE score ≥21)	15	5.12 ± 0.83
Moderate cognitive dysfunction (MMSE score of 10–20)	12	9.64 ± 1.35^a^
Severe cognitive dysfunction (MMSE score ≤9)	23	13.29 ± 2.38^ab^

*Note.* compared with patients with mild cognitive dysfunction, ^a^*P* < 0.05; compared with patients with mild and moderate cognitive dysfunction, ^b^*P* < 0.05.

The article "Changes in Levels of Homocysteine and C-Reactive Protein in Patients with Alzheimer's Disease and Their Correlation with Cognitive and UPDRS Functions" was retracted in 2023. Reasons: signs of a paper mill; suspected computer-generated content; unreliable results or conclusions; concerns about the data.

**Table 7:** Correlation analysis of patients' CRP with UPDRS scores ($\bar{x}$ ± *s*).

Class	Number of patients	Hcy (umol/L)
Total UPDRS score of 0∼20	12	5.26 ± 0.92
Total UPDRS score of 21∼40	17	9,76 ± 1.23^a^
Total UPDRS score of 41∼60	21	12.98 ± 3.23^ab^

*Note.* compared with patients with a total UPDRS score of 0∼20, ^a^*P* < 0.05; compared with the patients with a total score of 21∼40 and 41∼60, ^b^*P* < 0.05.

## Data Availability

The simulation experiment data used to support the findings of this study are available from the corresponding author upon request.
